This article has been retracted.

# Outcomes of Renal Stone Surgery Performed Either as Predonation or Ex Vivo Bench Procedure in Renal Grafts from Living Donors: A Systematic Review

**DOI:** 10.1155/2020/6625882

**Published:** 2020-11-27

**Authors:** Nicola Longo, Armando Calogero, Massimiliano Creta, Giuseppe Celentano, Luigi Napolitano, Marco Capece, Roberto La Rocca, Caterina Sagnelli, Nicola Carlomagno, Gaia Peluso, Teresa Pagano, Silvia Campanile, Concetta Anna Dodaro, Antonello Sica, Gianluigi Califano, Felice Crocetto, Ferdinando Fusco, Francesco Mangiapia, Michele Santangelo

**Affiliations:** ^1^Department of Neurosciences, Reproductive Sciences and Odontostomatology, University of Naples Federico II, 80131 Naples, Italy; ^2^Department of Advanced Biomedical Sciences, University of Naples Federico II, 80131 Naples, Italy; ^3^Department of Mental Health and Public Medicine, University of Campania Luigi Vanvitelli, 80131 Naples, Italy; ^4^Department of Precision Medicine, University of Campania Luigi Vanvitelli, 80131 Naples, Italy; ^5^Department of Woman, Child and General and Specialized Surgery, Urology Unit, University of Campania Luigi Vanvitelli, Naples, Italy

## Abstract

**Aims:**

We aimed to summarize available evidence about intraoperative and postoperative donors' and recipients' outcomes following stone surgery in renal grafts from living donors performed either before donation or as ex vivo bench surgery at the time of living-donor nephrectomy.

**Methods:**

A systematic review of PubMed, ISI Web of Knowledge, and Scopus databases was performed in September 2020. We included full papers that met the following criteria: original research, English language, human studies, and describing the results of stone surgery in renal grafts from living donors performed either before transplantation or as ex vivo bench surgery.

**Results:**

We identified 11 studies involving 106 patients aged between 22 and 72 years. Predonation and bench stone surgery was performed in 9 (8.5%) and 96 (90.6%) patients, respectively. Predonation stone surgery involved extracorporeal shock wave lithotripsy, retrograde intrarenal surgery, and percutaneous nephrolithotomy in 8, 1, and 1 patient, respectively. The overall success rate of predonation stone surgery was 78%, and the complication rate was 0%. Bench stone surgery involved ureteroscopy, pyelolithotomy, or a combination of both in 79 (82.3%), 10 (10.4%), and 7 (7.3%) cases, respectively, with an overall success rate of 95.8% and an overall complication rate of 9.37%.

**Conclusions:**

Predonation and bench stone surgery in grafts from living donors represents efficacious and safe procedures. Further studies on wider series with a longer follow-up are required.

## 1. Introduction

Renal transplantation (RT) from living donors provides significant advantages compared to transplantation from deceased donors including improved long-term survival, immediate functioning of the transplant, better transplant survival, and the possibility of transplanting preemptively [1–5]. An ideal kidney donor has no renal disease, no active infection, and no transmissible malignancy. Unfortunately, although the total number of kidney transplants has increased in the last years, the number of total living donations has remained stable with a subsequent decrease in the proportion of living donor transplant procedures [2]. Therefore, due to the shortage of living donors, centers have started using expanded criteria for donors, and RT from marginal donors has been proposed as a potential solution for organ shortage problems [6]. Historically, stone-bearing kidneys have not been accepted for transplantation in many institutions [7]. Indeed, stones located in the upper urinary tract of kidney donors represent a relative contraindication to RT because of complications like oliguria, hematuria, or rising creatinine in the receiver [8]. Moreover, the donor is exposed to the risk of future stone formation in the remaining kidney, which could lead to obstruction, infections, and end-stage renal disease [9]. Currently, the asymptomatic potential donor with a current single stone might be considered suitable for kidney donation in selected cases [10–12]. The need to cope with the living graft shortage together with the development of minimally invasive surgery and ex vivo bench surgery stimulated research toward the treatment of stones either in the pretransplantation setting or during back-table procedures [10]. In some institutions, the consideration of donors with stones has led to about 5% more RT than would otherwise have been possible [13]. Therefore, stone surgery in the donor's kidney before or during RT is expected to be carried out in an increasing number of cases in the next years. However, the optimal operative management for such patients is still under debate. The present review is aimed at summarizing available clinical evidence about the outcomes of stone surgery performed either in the predonation setting or as ex vivo bench surgery at the time of living-donor nephrectomy.

## 2. Evidence Acquisition

This analysis was conducted and reported according to the general guidelines recommended by the Primary Reporting Items for Systematic Reviews and Meta-analyses (PRISMA) statement [14]. To assess eligibility for the systematic review, PICOS (participants, intervention, comparisons, outcomes, study type) criteria were used [15]. PICOS criteria were set as follows: participants—living kidney donors with urolithiasis involving the kidney selected for donation; intervention—surgery for stones in kidney selected for donation performed either before RT or as ex vivo bench surgery at the time of living-donor nephrectomy; comparison—none; outcome—intra- and postoperative surgical outcomes; study type—prospective and retrospective studies and case reports. Three databases (PubMed, Scopus, and ISI Web of Knowledge) were searched for articles published in English up to August 2020. The following combinations of keywords were used to retrieve relevant articles: “renal transplantation” AND “living donor” AND “urolithiasis”. Abstracts (with no subsequent full-text publications) and articles that were not journal articles (letter, book, conference proceeding) or were not peer-reviewed studies were excluded. Two authors (GC and LN) reviewed the records separately to select relevant publications, with any discrepancies resolved by a third author (MC). The following data were extracted from the studies which included authors, year of publication, study period, study design, sample size, donors' age, gender, side of the kidney, stone size and location, type of surgery, operation time (OT), success of stone surgery, surgical complications during stone surgery, early (within 30 days) and late (>30 days) donors' and recipients' complications, grade of complication according to the Clavien-Dindo Classification System [16], recipients' age and gender, donors' and recipients' follow-up, and stone recurrence in the graft. The quality of the studies was assessed using the Newcastle–Ottawa scale (NOS) [17]. This scale measures three dimensions (selection, comparability of cohorts, and outcome). We rated the quality of the studies (good, fair, and poor) by awarding stars in each domain following the guidelines of the Newcastle–Ottawa Scale. A “good” quality score required 3 or 4 stars in selection, 1 or 2 stars in comparability, and 2 or 3 stars in outcomes. A “fair” quality score required 2 stars in selection, 1 or 2 stars in comparability, and 2 or 3 stars in outcomes. A “poor” quality score reflected 0 or 1 star(s) in selection, or 0 stars in comparability, or 0 or 1 star(s) in outcomes.

## 3. Results

The search strategy revealed 60 results. The screening of titles and abstracts revealed 18 full-text articles eligible for inclusion. Further assessment of eligibility, based on full-text papers, led to the exclusion of 7 papers. Finally, 11 studies involving 106 patients with a mean age ranging from 29.5 to 60 years who underwent stone surgery before or at RT from 1996 to 2020 were included in the final analysis (Figure 1) [8–11, 13, 18–23]. Specifically, seven studies (64%) were retrospective observational, two (18%) were prospective observational and two (18%) were case reports. The characteristics of the studies included as well as the features of donors and grafts are summarized in Table 1. The quality of the included studies is depicted in Table 2.

### 3.1. Predonation Stone Surgery

Overall, 9 (8.5%) patients underwent predonation stone surgery. Of them, 8 (88%), 1 (5%), and 1 (5%) underwent extracorporeal shockwave lithotripsy (ESWL), percutaneous lithotripsy (PCNL), and RIRS, respectively. Overall, these procedures were successful in 7 patients (78%). Intraoperative, early and late postoperative data about donors undergoing preoperative stone surgery and their recipients are reported in Table 3.

### 3.2. Bench Stone Surgery

Overall, ex vivo bench stone surgery was performed in 96 renal grafts. The surgical technique and the intraoperative outcomes are reported in Table 4. Bench ureteroscopy (URS), pyelolithotomy (PLT), and a combination of both were adopted in 79 (82.3%), 10 (10.4%), and 7 (7.3%) renal grafts, respectively. In patients undergoing bench URS, the access to the pyelocaliceal system was obtained through semirigid ureteroscopes, flexible ureteroscopes, and pediatric cystoscopes in 51 (53%), 35 (36.4%), and 8 (8.33%) cases, respectively. Stone fragmentation involved laser lithotripsy and pneumatic lithotripsy in 17 (17.7%) and 3 (3.12%) cases, respectively. Stone basketing alone was performed in 27 (28%) cases. The mean OT ranged from 1 to 49 minutes. Overall, bench procedures were successful in 92 (95.8%) cases and no complications were recorded. Early postoperative complications were recorded in 9 (9.37%) recipients. Mean recipients' follow-up ranged from 1 to 110 months. Late complications were recorded in 3 (3.1%) recipients. No stone recurrence in the graft was recorded. At a mean follow-up of 34.2 months (range: 1-110), no donors' complications were recorded.

## 4. Discussion

The selection of an appropriate living donor is critical for a successful RT. Given the improvements in minimally invasive renal surgery observed in recent years, attempts have been made to expand the donor pool by including so-called marginal living donors such as patients with small renal mass or urolithiasis [24, 25]. Urolithiasis affecting living kidney donors represents a significant challenge. Historically, patients wishing to donate their kidneys were deemed ineligible if preoperative imaging demonstrated nephrolithiasis due to the risk of complications that may be related to the stone itself or to the procedure of stone removal including infections, upper urinary tract obstruction, and graft loss [26]. The widespread use of computerized tomography angiography in the diagnostic workup of living donors has increased the detection of small asymptomatic renal stones with an incidence reaching up to 10% [27]. Subjects with small asymptomatic incidentally discovered stones represent a considerable percentage that might increase the donor pool [27, 28]. The guidelines developed in 1996 by the Ad Hoc Clinical Practice Guidelines Subcommittee of the Patient Care and Education Committee of the American Society of Transplant Physicians stated that “nephrolithiasis is at least a relative contraindication to living donor nephrectomy because of the future risk that recurrent stones, obstructions, and infections will injure the remaining kidney” and that “nephrolithiasis not only places the donor at risk; inadvertent transplantation of a kidney with stone places the recipient at risk” [29]. In 2004, kidney transplant physicians and surgeons met in Amsterdam for the International Forum on the Care of the Live Kidney Donor. During this forum, it was clearly stated that an asymptomatic potential donor with a current single stone might be considered suitable for kidney donation if (a) there is no hypercalciuria, hyperuricemia, or metabolic acidosis; (b) there is no cystinuria or hyperoxaluria; and (c) the current stone is <15 mm in size or potentially removable during transplant [12]. In a more recent nationwide survey, it has been shown that 84% of sharing institutions accepted patients with a history of nephrolithiasis [27, 30].

Once the decision to proceed with RT has been made, possible options include the donation of the non-stone-bearing kidney, donation of the stone-bearing kidney without stone removal, stone removal before RT, and bench stone removal at the time of RT [13].

Typically, the use of the stone-bearing kidney is preferred for donation because of the potential risk to the donor of obstruction from a stone in a solitary remaining kidney [13].

Surgical management of urolithiasis after RT represents a viable option. Indeed, several technological improvements have been introduced and are rapidly evolving to manage urolithiasis in a minimally invasive fashion in the general population as well as in patients who underwent RT [31–33]. Current European Association of Urology guidelines recommend considering conservative treatment for small asymptomatic stones only in absolutely compliant transplanted patients and to offer ESWL, flexible URS, and PCNL in other cases. Some authors propose a watchful waiting protocol for stones < 4 mm as the spontaneous stone-free rate in these cases varies between 60% and 100% [7, 11, 27, 34]. ESWL or antegrade/retrograde URS are strongly recommended for stones < 15 mm [32, 33]. Stone-free rates following ESWL vary between 40 and 80% and can reach 67% following URS. PCNL is recommended for stones > 20 mm, although the strength of the rating is weak [32, 33]. Overall, selecting the appropriate technique for stone removal in a transplanted kidney is difficult and stone surgery is more challenging when compared to nontransplanted patients [32, 33]. Moreover, the risk of surgery and stone-related complications could be significantly increased, mainly in recipients with increased comorbidity status [32, 33, 35].

Available technologies have made it possible to obtain stone clearance in the kidney from living donors either before donation or at the time of living-donor nephrectomy through bench surgery. To date, however, no clear recommendations exist about the operative management of urolithiasis in renal grafts from living donors.

The results from the present systematic review show that stone surgery is performed in living donors with mainly asymptomatic stones with a diameter ranging from 1 to 15 mm involving the whole pyelocalyceal system.

Operative management options include predonation stone surgery and ex vivo bench stone surgery. Criteria for selection of treatment modality have been reported by Ganpule et al. [20]. Authors treated hard stones with higher Hounsfield units (>1200) with ex vivo URS or PLT or preoperative RIRS with the choice between the two based on the pelvicalyceal anatomy (infundibular width, infundibular length, and pelvicalyceal angle) [20]. On the other hand, soft stones (<1200 Hounsfield units) were managed with pretransplant ESWL performed with low energy, frequency, and power parameters [20]. Most published series describe grafts treated through ex vivo bench surgery, and therefore, it represents the recommended treatment option for stones < 15 mm in size or potentially removable during RT [11, 12, 27]. Potential advantages of ex vivo bench procedures include reduced donors' morbidity, shorter waiting times for donation, and lower costs [21]. Ex vivo bench removal of upper urinary tract stones may be achieved by URS, PLT, basket retrieval, or a combination of them. The choice of surgical procedure depends on the size and location of stones. Available literature shows that URS represents the preferred option in most cases. Great diversity in the methods of bench URS exists that mostly reflects the wide variety of surgical devices used. Indeed, the procedure may be performed with cystoscopes and semirigid and flexible ureteroscopes. Moreover, stone clearance may be obtained through forceps, pneumatic, or laser lithotripsy. Finally, baskets can be used for the extraction of stones or fragments [27]. Semirigid ureteroscopes are preferred over flexible ones for bench URS because of easier handling [22]. Indeed, most calyces can be accessed on the bench using a semirigid scope due to ureteral mobility [22]. Flexible scopes are useful when a stone needs to be extracted from a lower calyx with acute angulation [22]. Pediatric cystoscopes have the advantage of better stability and maneuverability due to the short length of the shaft [20]. Holmium laser is considered a better option than pneumatic energy thanks to the lower risk of mucosal injury in a kidney that is completely flaccid with a stone that lacks firm support [22]. PLT is considered by some authors an excellent method for extracting intact stones during bench surgery mainly in the case of the extrarenal pelvis [22]. It can be performed in combination with URS for stone extraction or if the ureter is tight [20]. OT represents a critical variable to be addressed. Indeed, cold ischemia time > 8 h can potentially jeopardize renal function, increase acute rejection rates, or affect long-term graft survival [11]. Interestingly, the mean OT reported by most available studies was within 30 minutes. Opinions about the technical complexity of bench stone surgery are controversial. Pushkar et al. consider bench URS a challenging procedure to be done by expert hands only as the kidney is unstable and avascular, and the intrarenal orientation can change with movements [22]. Other authors consider bench surgery an easy-to-learn procedure with a short learning curve, as it is easier to handle and maneuver the kidney on the back table [11, 13]. The success rate with bench procedures is high in most series. Surgical failures may be due to anatomical abnormalities [22]. For example, if stones are located in calyces with narrow infundibulum, they can be left in situ and transplantation can proceed as the risk of stone dislodgement is negligible [22]. RT represents a complex surgical procedure that may be associated with several medical and surgical complications [36–39]. Predonation and bench stone surgery may potentially increase the complication rate of RT both in the early and late postoperative stages.

Interestingly, none of the recipients who received graft from living donors undergoing predonation stone surgery reported early postoperative complications.

Short-term concerns with bench surgery include ureteric injury, hematuria, urine leak, and graft dysfunction [22]. Notably, evidence demonstrates a low incidence of short-term complications in recipients of grafts undergoing bench stone surgery. Indeed, early postoperative complications were recorded in 9 cases and in only two cases, these complications were attributed to bench stone surgery. One patient developed a urinary leakage after PLT that was repaired with primary suture [11]. The second one involved a complete occlusion of the ureteroneocystostomy after bench URS and was treated with exploration and revision of the ureteroneocystostomy [23].

Several risk-reduction strategies have been proposed to prevent ureteral injury during ex vivo endourologic manipulations: minimal handling of the ureter, a minimum influx of irrigant fluid to prevent the potential for pyelovenous and pyelolymphatic backflow, adoption of small instruments, and placement of a double-J ureteral stent [20].

Stone recurrence in grafts is a potential long-term concern. Of note, none of the grafts undergoing stone surgery showed evidence of stone recurrence at the follow-up examination.

Taken together, data synthesized in the present review support the role predonation and bench stone surgery in the case of urolithiasis involving renal grafts from living donors and emphasize the feasibility to extend the pool of living donors to subjects with stone bearing kidneys.

However, potential limits of available literature must be acknowledged: available studies are few, of low methodological quality, and with short follow-up. They enroll a small number of patients, and often, populations and surgical techniques employed are different. Moreover, only a few studies reported complications according to the Clavien-Dindo Classification System. Therefore, available level of evidence is low and still inadequate to provide definitive recommendations. Further well-designed studies on wider series with long-term follow-up are strongly advocated to confirm these preliminary data.

## 5. Conclusions

Surgical treatment of urolithiasis in kidney grafts from living donors can be efficiently and safely addressed through both predonation and ex vivo bench procedures. These procedures are associated with a high success rate and low complication rate. No cases of stone recurrence in the graft have been reported. Data from larger studies with long-term follow-up are advocated.

## Figures and Tables

**Figure 1:** Flow diagram of the systematic review.

**Table 1:** Study features and baseline characteristics of living kidney donors and recipients.

Author, year of publication	Study period	Study design	Sample size (*n*)	Donor's age (years), mean (range)	Donor's gender M : F	Graft side Ri : Le	Stone location (n)	Stone size, mm mean (range)	Recipient's age (years), mean (range)	Recipient's gender M : F
Rashid et al., [18]	1996-2000	R	10	45.0 (27-58)	4 : 6	n/a	3^uc^ 3^mc^ 4^lc^	5.2 (1-8)	41.5 (18-72)	6 : 4
Yiğit et al., [21]	1999-2003	P	2	29.5 (30-49)	2 : 0	n/a	n/a	6.0 (5-7)	n/a	n/a
Trivedi et al., [19]	2007	CR	1	n/a	n/a	n/a	1^lc^	5.0 (n/a)	n/a	n/a
Schade et al.,[23]	1996-2010	R	23	44.0 (24-67)	8 : 15	n/a	5^uc^ 10^mc^ 13^lc^	3.9 (3-6)	41.5 (3-72)	13 : 10
Vasdev et al.,[9]	2004-2008	R	3	47.6 (46-50)	n/a	0 : 3	1^mc^ 2^lc^	3.6 (3-5)	29.3 (22–51)	n/a
Olsburgh et al., [13]	2005-2011	R	17	45.0 (22-67)	n/a	8 : 12	5^uc^ 5^mc^ 10^lc^	2.5 (2-12)	39.0 (1-66)	n/a
Ganpule et al., [20]	n/a	R	12	52.3 (38-71)	4 : 8	3 : 3	2^mc^ 5^lc^	4.9 (1.8-6)	n/a	n/a
Pushkar et al., [22]	2013-2014	P	14	44.8 (27-64)	5 : 9	4 : 10	7^uc^ 5^mc^ 4^lc^	6.3 (4-10)	n/a	n/a
Lin et al., [10]	2010-2015	R	10	48.8 (28-58)	4 : 6	0 : 10	1^uc^ 3^mc^ 6^lc^	5.8 (2-9)	n/a	n/a
Sarier et al., [11]	2009-2016	R	13	52.3 (40-72)	6 : 7	n/a	3^uc^ 5^mc^ 4^lc^ 1^p^	9.1 (5-15)	n/a	n/a
Barki et al., [8]	2020	CR	1	60.0 (n/a)	0 : 1	0 : 1	1^uc^	9.0 (n/a)	22.0 (n/a)	1 : 0

CR: case report; F: female; Le: left; M: male; n/a: not available; P: prospective; R: retrospective; Ri: right; ^uc^Upper calyx; ^mc^middle calyx; ^lc^lower calyx; ^p^pelvis.

**Table 2:** Risk of bias assessment based on the Newcastle–Ottawa Quality Assessment Scale criteria.

Study	Selection	Comparability	Outcome	Total score	Quality score
Rashid et al., [18]	★ ★	—	★	★ ★ ★	Poor
Yiğit, [21]	★★	—	★	★ ★ ★	Poor
Trivedi et al., [19]	—	—	★	★	Poor
Schade et al., [23]	★ ★ ★	—	★ ★	★ ★ ★ ★ ★	Poor
Vasdev et al., [9]	★★	—	★ ★	★ ★ ★ ★	Poor
Olsburgh et al., [13]	★ ★ ★	—	★	★ ★ ★ ★	Poor
Ganpule et al., [20]	★ ★ ★	—	★	★ ★ ★ ★	Poor
Pushkar et al., [22]	★ ★ ★	—	★	★ ★ ★ ★	Poor
Lin et al., [10]	★ ★	—	★	★ ★ ★	Poor
Sarier et al., [11]	★ ★ ★	★ ★	★ ★	★ ★ ★ ★ ★ ★ ★	Good
Barki et al., [8]	—	—	★	★	Poor

**Table 3:** Predonation stone surgery: donors' and recipients' outcomes.

	Donors' outcomes						Recipients' outcomes		
Author, year of publication	Surgery type (*n*)	OT min, mean (range)	Success : failed	Early postoperative complication type, *n* (grade^∗^)	Follow-up (months) (range)	Late postoperative complication type, *n*	Early postoperative complication type, *n* (grade^∗^)	Follow-up (months) (range)	Stone recurrence in the graft (*n*)
Yiğit et al., [21]	ESWL (2)	n/a	1 : 1	0 (-)	n/a	n/a	0 (-)	6.0 (n/a)	0
Trivedi et al., [19]	ESWL (1) PCNL (1)	n/a	0 : 1	0 (-)	n/a	0	0 (-)	24 (n/a)	0
Ganpule et al., [20]	ESWL (5) RIRS (1)	n/a	6 : 0	0 (-)	36.0 (10-58)	0	0 (-)	36.0 (10-58)	0

ESWL: extracorporeal shock wave lithotripsy; n/a: not available; OT: operative time; PCNL: percutaneous nephrolithotomy; RIRS: retrograde intrarenal surgery. ^∗^According to the Clavien-Dindo Classification System.

**Table 4:** Bench stone surgery: technique and outcomes.

Author, year of publication	Type of surgery (*n*)	Instrumentation for access to the pyelocaliceal system type (*n*)	Instrumentation for stone fragmentation/extraction type (*n*)	OT min, mean (range)	Success : failed	Bench surgery complication, type (*n*)	Donors' follow-up (months), mean (range)	Donors' late postoperative complications (*n*)	Recipients' early postoperative complication type, *n* (grade^∗^)	Recipients' follow-up (months), mean (range)	Recipients' late postoperative complication type (*n*)	Stone recurrence in the graft (*n*)
Rashid et al., [18]	URS (10)	6.9 Fr su (9) 9.5 Fr fu (1)	Holmium laser lithotripsy (6) Basketing (3) Negative ureteroscopy (1)	6.5 (3-28)	10 : 0	0	36.4 (8-60)	0	0	33.2 (18-60)	Ischemic fistula (1)	0
Yiğit et al., [21]	PLT (1)	n/a	n/a	n/a	1 : 0	0	n/a	0	0	n/a	n/a	0
Trivedi et al., [19]	URS (1)	8.5 Fr su (1)	Pneumatic+forceps (1)	n/a	1 : 0	0	n/a	0	0	24.0 (n/a)	0	0
Schade et al., [23]	URS (23)	6.9 Fr su (21) 9.5 Fr fu (2)	Holmium laser lithotripsy (6) Basketing (12) Negative ureteroscopy (4)	6.2 (3-16)	22 : 1	0	63.0 (n/a)	n/a	Ureteroneocystostomy stenosis, 1 (n/a) Wound cellulitis, 1 (II) Lymphocele, 3 (>II) Death, 1 (V)	63.0 (16-110)	Transplant nephrectomy (1) Hemodialysis (1)	0
Vasdev et al., [9]	URS (3)	7.5 Fr fu (3)	Basketing (3)	n/a	3 : 0	0	64.0 (48-84)	0	0	64.0 (48-84)	0	0
Olsburgh et al., [13]	URS (17)	7.5 Fr fu (17)	Holmium laser lithotripsy (4) Basketing (5) Laser and basketing (1) Negative ureteroscopy (6)	n/a (10-45)	16 : 1	0	26.0 (12-49)	0	0	10.0 (1-24)	0	0
Ganpule et al., [20]	URS (1)	6 Fr pc (1)	Basketing (1)	20.0 (n/a)	3 : 0	0	36.0 (10-58)	0	0	36.0 (10-58)	0	0
	PLT (2)	12 Fr nephroscope (2)	Basketing (2)	n/a								
Pushkar et al., [22]	URS (7) URS+PLT (7)	6/7.5 Fr su (11) 5.3 Fr fu (3)	Laser+basketing (3) Pneumatic+forceps (2) Basket only (1)	28.0 (22-49)	13 : 1	0	12.0 (6-18)	0	Mild graft dysfunction, 2 (n/a)	16.0 (12-24)	0	0
Sarier et al., [11]	URS (6)	6/7.5 Fr su (6) 7.5 Fr fu (1) 8/9.8 Fr 12° pc (6)	Laser and basketing (6)	12.5 (9-20)	12 : 1	0	0	n/a	0	49.6 (14-101)	0	0
	PLT (7)	8/9.8 Fr 12° pc (1)	Laser and basketing (1)	3.1 (1-8)					Urinary leakage, 1 (IIIb)			
Lin et al., [10]	URS (10)	6.5/8.5 Fr su (3) 6.5/8.5 Fr fu (7)	Forceps (3) Laser+basketing (7)	21.2 (14-31)	10 : 0	0	12.0 (n/a)	0	0	12.0 (n/a)	0	0
Barki et al., [8]	URS (1)	fu (1)	Laser (1)	17.0 (n/a)	1 : 0	n/a	n/a	n/a	n/a	n/a	n/a	n/a

Fr: French; fu: flexible ureteroscope; OT: operative time; pc: pediatric cystoscope; PLT: pyelolithotomy; su: semirigid ureteroscope; URS: ureteroscopy. ^∗^According to the Clavien-Dindo Classification System.

## Data Availability

No data were used to support this study.

## References

[1] Dols L. F. C., Kok N. F. M., IJzermans J. N. M. (2010). Live donor nephrectomy: a review of evidence for surgical techniques. *Transplant International*.

[2] Lee L. Y., Pham T. A., Melcher M. L. (2019). Living kidney donation: strategies to increase the donor pool. *The Surgical Clinics of North America*.

[3] Hart A., Smith J. M., Skeans M. A. (2018). OPTN/SRTR 2016 annual data report: kidney. *American Journal of Transplantation*.

[4] Creta M., Calogero A., Sagnelli C. (2019). Donor and recipient outcomes following robotic-assisted laparoscopic living donor nephrectomy: a systematic review. *BioMed Research International*.

[5] Calogero A., Sagnelli C., Peluso G. (2020). Physical activity in elderly kidney transplant patients with multiple renal arteries. *Medicine & Pharmacology*.

[6] Hamano I., Hatakeyama S., Fujita T. (2020). Living kidney transplantation from marginal donors presents feasible donor renal function despite inferior recipient renal function. *Transplantation Proceedings*.

[7] Devasia A., Chacko N., Gnanaraj L., Cherian R., Gopalakrishnan G. (2005). Stone-bearing live-donor kidneys for transplantation. *BJU International*.

[8] Barki A., Mhanna T., Aynaou M., Chennoufi M., Boateng P. d., Houmaidi A. E. L. (2020). *Ex vivo* treatment of stones in living donor kidney by flexible ureteroscopy: time challenge (case report). *Urology Case Reports*.

[9] Vasdev N., Moir J., Dosani M. T. (2011). Endourological management of urolithiasis in donor kidneys prior to renal transplant. *ISRN Urology*.

[10] Lin C. H., Zhang Z. F., Wang J. (2017). Application of ureterorenoscope and flexible ureterorenoscope lithotripsy in removing calculus from extracorporeal living donor renal graft: a single-center experience. *Renal Failure*.

[11] Sarier M., Duman I., Yuksel Y. (2018). Ex vivo stone surgery in donor kidneys at renal transplantation. *International Journal of Urology*.

[12] Delmonico F., Council of the Transplantation Society (2005). A report of the Amsterdam forum on the care of the live kidney donor: data and medical guidelines. *Transplantation*.

[13] Olsburgh J., Thomas K., Wong K. (2013). Incidental renal stones in potential live kidney donors: prevalence, assessment and donation, including role of ex vivo ureteroscopy. *BJU International*.

[14] Liberati A., Altman D. G., Tetzlaff J. (2009). The PRISMA statement for reporting systematic reviews and meta-analyses of studies that evaluate health care interventions: explanation and elaboration. *Annals of Internal Medicine*.

[15] Schardt C., Adams M. B., Owens T., Keitz S., Fontelo P. (2007). Utilization of the PICO framework to improve searching PubMed for clinical questions. *BMC Medical Informatics and Decision Making*.

[16] Clavien P. A., Barkun J., de Oliveira M. L. (2009). The Clavien-Dindo classification of surgical complications. *Annals of Surgery*.

[17] Stang A. (2010). Critical evaluation of the Newcastle-Ottawa scale for the assessment of the quality of nonrandomized studies in meta-analyses. *European Journal of Epidemiology*.

[18] Rashid M. G., Konnak J. W., Wolf J. S. (2004). Ex vivo ureteroscopic treatment of calculi in donor kidneys at renal transplantation. *The Journal of Urology*.

[19] Trivedi A., Patel S., Devra A., Rizvi J., Goel R., Modi P. (2007). Management of calculi in a donor kidney. *Transplantation Proceedings*.

[20] Ganpule A., Vyas J. B., Sheladia C. (2013). Management of urolithiasis in live-related kidney donors. *Journal of Endourology*.

[21] Yiğit B., Aydin C., Titiz I., Berber I., Sinanoğlu O., Altaca G. (2004). Stone disease in kidney transplantation. *Transplantation Proceedings*.

[22] Pushkar P., Agarwal A., Kumar S., Guleria S. (2015). Endourological management of live donors with urolithiasis at the time of donor nephrectomy: a single center experience. *International Urology and Nephrology*.

[23] Schade G. R., Stuart Wolf J., Faerber G. J. (2011). *Ex-vivo* ureteroscopy at the time of live donor nephrectomy. *Journal of Endourology*.

[24] Lim S. Y., Kim M. G., Park K. T., Jung C. W. (2017). Experiences of renal transplants from donors with renal cell carcinoma after ex vivo partial nephrectomy. *Annals of Surgical Treatment and Research*.

[25] Schiavina R., Mari A., Antonelli A. (2015). A snapshot of nephron-sparing surgery in Italy: a prospective, multicenter report on clinical and perioperative outcomes (the RECORd 1 project). *European Journal of Surgical Oncology*.

[26] Rizkala E., Coleman S., Tran C. (2013). Stone disease in living-related renal donors: long-term outcomes for transplant donors and recipients. *Journal of Endourology*.

[27] Harraz A. M., Kamal A. I., Shokeir A. A. (2016). Urolithiasis in renal transplant donors and recipients: An update. *International Journal of Surgery*.

[28] Kamal A. I., Harraz A. M., Shokeir A. A. (2011). Controversies related to living kidney donors. *Arab Journal of Urology*.

[29] Kasiske B. L., Ravenscraft M., Ramos E. L., Gaston R. S., Bia M. J., Danovitch G. M. (1996). The evaluation of living renal transplant donors: clinical practice guidelines. Ad Hoc Clinical Practice guidelines Subcommittee of the Patient Care and Education Committee of the American Society of Transplant Physicians. *Journal of the American Society of Nephrology*.

[30] Brar A., Jindal R. M., Abbott K. C., Hurst F. P., Salifu M. O. (2012). Practice patterns in evaluation of living kidney donors in United Network for Organ Sharing-approved kidney transplant centers. *American Journal of Nephrology*.

[31] Barone B., Crocetto F., Vitale R. (2020). Retrograde intra renal surgery versus percutaneous nephrolithotomy for renal stones >2 cm. A systematic review and meta-analysis. *Minerva Urologica e Nefrologica*.

[32] Türk C., Neisius A., Petrik A. (2020). EAU guidelines on urolithiasis. *EAU guidelines*.

[33] Breda A., Budde K., Figueiredo A., Lledó García E., Olsburgh J., Regele H. (2020). *EAU guidelines on renal transplantation*.

[34] Martin G., Sundaram C. P., Sharfuddin A., Govani M. (2007). Asymptomatic urolithiasis in living donor transplant kidneys: initial results. *Urology*.

[35] Calogero A., Sagnelli E., Creta M. (2019). Eradication of HCV infection with the direct-acting antiviral therapy in renal allograft recipients. *BioMed Research International*.

[36] Peluso G., Incollingo P., Campanile S. (2020). Relation between wound complication and lymphocele after kidney transplantation: a monocentric study. *Transplantation Proceedings*.

[37] Scotti A., Santangelo M., Federico S. (2014). Complicated diverticulitis in kidney transplanted patients: analysis of 717 cases. *Transplantation Proceedings*.

[38] Calogero A., Gallo M., Sica A. (2020). Gastroenterological complications in kidney transplant patients. *Open Medicine*.

[39] Mirone V., Longo N., Fusco F. (2009). Renal transplantation does not improve erectile function in hemodialysed patients. *European Urology*.

